RETRACTED

# Human-Computer Interaction Environment Monitoring and Collaborative Translation Mode Exploration Using Artificial Intelligence Technology

**DOI:** 10.1155/2022/4702003

**Published:** 2022-09-30

**Authors:** Yunzhi Shao

**Affiliations:** Yangzhou Polytechnic College, Jiangsu, Yangzhou 225009, China

## Abstract

Artificial intelligence now plays a significant role in both daily life and scientific research because of the rapid advancement of this technology in recent years. Making full use of the phrases in the translation phrase table for translation is challenging since the phrase matching is too accurate when the translation machine decodes. Fully automatic machine translation struggles to meet the expectations of its users since there are more or less translation faults brought on by data bottlenecks. Therefore, we require collaborative assisted translation technology for human-computer interaction. This work strengthens the research on collaborative translation techniques and ways for monitoring the human-computer interaction environment in order to further improve translation quality. This essay investigates and discusses human-computer translation techniques as well as related ideas in collaborative translation and human-computer interaction. The translation similarity model is incorporated into the translation system model together with an overall qualitative knowledge and logical reasoning capability of human-computer interaction to offer fresh strategies and methods for collaborative translation between humans and computers. According to the experimental findings, the accuracy rate of the collaborative translation system for human-computer interaction based on artificial intelligence technology can achieve 98.2% and 95.6%. The quality of the translation is enhanced after human-computer interaction, and the editing gap between the incorrect and auxiliary translations is narrowed, demonstrating the efficiency of the system and demonstrating its viability. In order to enhance the accuracy of system translation and the effectiveness of system operation, it is important to investigate the collaborative translation mode of human-computer interaction based on artificial intelligence technology.

## 1. Introduction

Artificial intelligence now plays a significant role in both daily life and scientific research because of the rapid advancement of this technology in recent years. Interaction design can realize “What you think is what you get,” “What you use is what you see,” and “What you see is what you hear” through artificial intelligence. Artificial intelligence technology combines user experience and evaluation closely through the analysis of user interaction behavior patterns and the reasoning of mental models and perceptual cognitive logic, thus changing the feedforward and feedback of interaction and ultimately affecting interaction design methods. In addition to altering the way people interact with computers, artificial intelligence technology also undermines the established human-computer relationship. As a result, the question of how to integrate artificial intelligence technology into interaction design has gained significant importance [1]. Artificial intelligence technology's explosive growth in 2016 has sparked a broad technological revolution across several industries. It is now possible to examine the human thinking style on the basis of having a more effective machine learning model and massive data processing capabilities [2]. We may employ artificial intelligence technology in interface design to give users a more natural and better interaction because it has entirely transformed the way and method of human-computer interaction [3]. Although learning is a complex process in the human thought process, it is also full with rules to abide by. Modern educational theory research has made judging a person's behaviour pattern through an examination of his or her learning preferences and thought patterns, followed by directional training and correction, a key component. The advancement of machine translation technology is a sign of the advancement of cognitive science, thinking science, and artificial intelligence [4, 5], and the introduction of certain effective translation systems will greatly advance society. Therefore, there is a lot of theoretical relevance and practical usefulness in the development and application of machine translation technology. Machine translation technology has achieved significant advancements over the past 50 years thanks to the constant advancement of artificial intelligence research and the widespread use of intelligent systems [6]. It has also become one of the major components of the entire area of study.

RETRACTED

More and more individuals are relying on the machine translation system as the quality of the translations is improving. We need a human-computer interactive collaborative assisted translation technology [7] because the issue of phrase matching being too accurate when the translation machine decodes makes it difficult to use the phrases in the translation phrase table for translation, and the translation errors caused by more or less data bottlenecks in automatic machine translation make the translation quality difficult to meet people's needs for translation. Human intervention mechanism is adopted to provide users with satisfactory translation results. Due to the diversity and complexity of language phenomena, after decades of exploration and research, the fully automatic machine translation system is still difficult to meet the practical requirements in many fields, and the quality of the translation is still unacceptable to people. It needs to spend a lot of time on manual postediting of the machine translation, and the gains outweigh the losses [8]. Therefore, people begin to realize that it is more practical to study how to realize human-machine symbiosis and human-machine mutual assistance in machine translation, instead of blindly pursuing fully automatic high-quality translation. Computer human-computer collaborative translation technology came into being [9]. The computer provides help to translators through electronic dictionaries, terminology management, translation memory, and other tools, greatly reducing repetitive work, reducing labor intensity, and improving the translation level of translators. In addition to using their professional expertise and common sense to guarantee that the translation is accurate, translators may also help the translation system perform better by providing feedback information [10]. Together, they advance in their work and learn from one another. Translation technology has advanced significantly after many years of development. Through the interaction mode offered by the human-machine interface, the collaborative translation system for human-machine interaction can address issues that are challenging to address by depending solely on the machine translation system. For example, the troublesome ambiguity phenomena including syntax, grammar, word meaning, and even context can make the user operate the system in a very natural and intuitive manner, making the system easy to master and use, and the knowledge level of the user is not high, all kinds of users can use [11].

Therefore, it is essential to investigate the cooperative translation method of human-computer interaction based on artificial intelligence technology. Therefore, this work has enhanced the research on collaborative translation methodologies and forms of human-computer interaction in order to further improve translation quality. This essay investigates and discusses human-computer translation techniques as well as related ideas in collaborative translation and human-computer interaction. A collaborative translation model system based on human-computer interaction is suggested to increase the English-Chinese translation system's translation accuracy. The translation similarity model is added to the translation system model together with a general qualitative grasp of human-computer interaction and the capacity for logical reasoning. The English-Chinese translation results can be produced by computing the translation similarity between two semantic vectors in the same semantic space, which offers a new technique and strategy for collaborative translation and human-computer interaction.

RETRACTED

The design of the suggested human-computer interaction collaborative translation system is studied in light of the investigation of human-computer collaborative translation mode based on artificial intelligence technology. The primary contributions and innovations of this paper are as follows:

1. The phrase table is simplified by this technology. The basic idea is as follows: if a phrase appears more frequently in several longer phrases, then this phrase is the information that plays a key role in translation; if a long phrase and its subphrase appear at the same frequency, then the long and short phrases may play a greater role in translation; if a phrase often appears in a longer phrase and rarely appears alone, it is likely that the phrase appears frequently but is not very useful for translation
2. This paper proposes a method of word selection based on user's translation history. After the translation template is determined, the variable part in the template needs to be translated. For the case that the same word or phrase has many different translation methods, this paper determines the choice of word meaning by calculating the similarity between all sentences containing the variable in the current user's translation history and the current sentence to be translated
3. An automatic postediting technology based on machine translation is proposed. The machine translation is taken as the source language, and the correct translation modified by each user is taken as the target language. The statistical translation model is trained by the human-computer interaction collaborative system. Before recommending the machine translation to the current user, the machine translation is translated into an auxiliary translation closer to the correct translation by its own translation model. Thus, the number of postediting operations by the user can be further reduced, and the efficiency of collaborative translation can be improved

## 2. Related Work

Collaboration refers to the process or ability to coordinate two or more resources or individuals to jointly complete a task or achieve a goal. The deepening of information technology, the improvement of computer computing ability, and the development of computer network technology have opened a new page for collaborative technology. Casa Kubeta proposed a collaborative translation mode and system framework with word segments as granularity units. The system fully exploits the advantages and traits of both humans and computers, allowing users and machine translation to be effectively coordinated and controlled. Additionally, various translational data are sensibly analysed and stored, increasing the system's translation efficiency and quality [12]. Anastasiou and Gupta believe that the field of machine translation has greatly deepened people's understanding of language, knowledge, intelligence, and other issues and promoted the development of related disciplines. The earliest machine translation was based on simple word translation, word frequency statistics, and word order changes. When people realized the limitations of this method, they began to strengthen the analysis of natural language understanding [13]. Nguyen et al. proposed the idea of collaborative translation based on user model. In the process of translation, the system provides users with dictionary, translation memory, terminology management, and other help and collects and records users' translation behavior in real time. By analyzing the user's behavior attribute and state attribute, the system creates a user model, and recommends more appropriate auxiliary translations for them. The user delivers its feedback knowledge to the system, which improves the performance of the system and enables users to dynamically share translation knowledge and implement online collaborative work. In this process, the knowledge has been effectively circulated, the translation knowledge of users and the system has been jointly enhanced, and the translation ability of both is constantly improved [14]. Makin et al. ensure the smoothness of the translation by modifying the machine translation, and the machine translation engine translates the translation back to the source language. The proposed system gives full play to the different roles of monolingual users of the two languages in translation [15]. Shailesh et al. designed an English-Chinese translation system based on variational model. Combining the variational algorithm and the adversarial neural network, calculate the Bleu value of the variational adversarial neural network translation, train the corpus data, and complete the design of the English-Chinese translation system [16] Anastasio and Gupta believe that if some machine translation systems can be defined or selected by human, the accuracy and quality of machine translation can be greatly improved. In general, machine translation has not reached the level where it can replace professional translation [17]. Hashimoto et al. described an online collaborative translation system for monolingual users. The system can enable monolingual users in the source language and the target language to perform collaborative translation online and make a clear division of labor between the two. The correctness of the translation is ensured by comparing whether the source language sentence newly generated by the translation engine is the same as the original sentence [18].

RETRACTED

From the research results listed above, the research on human-computer interaction and collaborative translation mainly focuses on two aspects: ① human-computer interaction, that is, how to coordinate and control people and computers and how to reasonably store various data so as to improve the quality and efficiency of translation; ② how to build an online collaborative translation environment and organize experts with various knowledge to complete a translation task together. The disadvantage is that different users have different translation habits and needs. Although some scholars have started to explore this field, the research is not extensive, in-depth, and specific. At the level of theoretical research, it still has many unsatisfactory places and needs further development and improvement. The research results of relevant scholars on the exploration of human-computer interaction collaborative translation mode based on artificial intelligence technology are less involved. As a result, the author is of the opinion that the investigation of collaborative translation mode based on artificial intelligence technology has some potential application value. This study analyses the machine translation system using an overview of traditional human-computer collaborative translation as well as the state-of-the-art background of artificial intelligence technology. Finally, an experimental study of the system is conducted, which significantly aids it in enhancing translation quality going forward.

## 3. Methodology

### 3.1. Human-Computer Interaction and Collaborative Translation

#### 3.1.1. Related Concepts of Traditional Human-Computer Interaction and Collaborative Translation

In order for the computer to carry out the conversion of the input source language into the appropriate target language and the translated result language in accordance with the algorithms, machine translation involves converting the laws of human natural language translation into computer algorithms. In this technique, humans employ the computer's quick processing power to assist them in translating papers. A crucial phase in the development of machine translation is collaborative translation and human-computer interaction. Human-computer interaction (HCI) is the process of merging computers and people in order to fully use the logical reasoning capabilities of computers and the general qualitative cognitive capabilities of humans. The left to right interaction framework is used in conventional interactive machine translation [19]. In the human-computer interaction framework, given a sentence in the source language to be translated, the user can perform translation completion or error correction from left to right. The system provides completion suggestions for subsequent translation according to the correct translation prefix confirmed by the user. Key errors refer to translation errors that have a great impact on the translation quality of other words or phrases in a sentence. Critical errors are often caused by the inherent difficulties in translating source side phrases [20]. The collaborative translation of human-computer interaction mainly ensures that the translation system can correctly translate the input content through the preprocessing of translation. The general process is as follows: after the source language sentence is input into the translation system, the translation system will segment all the phrases in the source language sentence and then compare the phrase sequence. If all the phrases are in the phrase table, the translation will be directly performed and the translation result will be output. If the phrases are not all in the phrase table, the phrase fuzzy matching is used to expand and translate the sentences. Then, the combined classifier is used to select the translation result with improved translation quality. Finally, the final translation result is selected by human judgment and output.

RETRACTED

The well-known machine translation pyramid provides a summary of the level of knowledge used in the machine translation model as well as the state of knowledge application for the statistical machine translation model as of the present. The best translation should take the word-level information of the source language and further turn it into the word order of the destination language, resulting in an intermediate language framework.  Figure 1 depicts the conceptual diagram of the machine translation pyramid.

According to Figure 1, there are three general categories into which statistical machine translation models fall: word-based translation models, phrase-based translation models, and syntax-based translation models. Three types of models can be distinguished among them, based on the differences in the degree of syntactic processing between the source language and the destination language: string to tree models, tree to string models, and tree to tree models. Generally speaking, regardless of whether it is a word-based translation model or a syntax-based translation model, each word in the source language sentence is individually translated into a word of the target language, even though different generation processes are used to explain how to adjust the word order of the target language.

RETRACTED

The application of human-computer interaction in machine translation can be described as correcting errors in speech recognition results through various interaction modes between human and machine. This is actually a kind of preprocessing before translation, which can only ensure that the translation system has completely correct input, and is not helpful to solve the difficulties of translation itself. In the process of translation, we should not rely on the machine to solve all problems, but should cooperate with the machine to complete the translation task.

#### 3.1.2. Correlation Analysis of Machine Translation System

With the rapid growth of the scale of translation tasks, it has to be completed by several, dozens, or even more translators. In the same task, many identical or similar documents, sentences, and terms will appear repeatedly. People can not help but think of applying collaborative technology to translation, to avoid repetitive translation content, reduce certain workload, and improve translation efficiency. Therefore, many translators are organized in different forms to complete the translation of various texts, that is, collaborative translation. Manual intervention: there are four methods as follows: ① preediting, ② interactive intervention, ③ postediting, and ④ manual translation of sentences rejected by the system. Among them, “the sentences rejected by the system are translated manually” is adopted by all practical systems. For preediting, the user must be clear about the system's restrictions on the translated original. For postediting, the user must master foreign languages. For manual interactive intervention, when the system encounters ambiguity and cannot be solved, it will send a query to the user and continue after the user answers. Questions and answers are given by the user's mother tongue, so the user does not need to master foreign languages and comply with too many restrictions of the system.

According to different research methods, machine translation can be divided into two categories: rationalism-based method and empiricism-based method. The method based on rationalism describes language in a certain form and summarizes language phenomena. It can also be called rule-based method, mainly including machine translation based on transformation, machine translation based on intermediate language, and machine translation based on knowledge. Empirical-based methods mainly include case-based machine translation and statistical-based machine translation. Template-based machine translation is the combination and optimization of rule-based and case-based machine translation. Compared with the rule-based method, template-based machine translation includes variables and a large number of specific content, which avoids the disadvantages of too abstract and error prone rule representation. Compared with the case-based method, because there are some variables in the template-based machine translation, it can cover more language phenomena than the case-based method in the same corpus, unlike the case-based method, which needs to maintain a huge case base. The translation template consists of two parts: the source language template and the target language template. Each part is composed of a frame and a slot. A frame is a fixed part of a template and consists of constants, that is, words or phrases.

RETRACTED

### 3.2. Design of Human-Computer Interaction Collaborative Translation System Based on Artificial Intelligence Technology

To address the demands of acquiring high-quality translation while gaining high-efficiency machine translation, a collaborative interactive human-machine translation system was designed.  Figure 2 depicts the human-computer interaction module of the artificial intelligence-based human-computer collaborative translation system.

The human-computer interactive collaborative translation system based on artificial intelligence technology is composed of graphical interface, indicator loading, indicator calculation, translation, and translation quality evaluation and other modules. For the function of graphical interface, human-computer interaction interface can be provided, such as loading sentences to be translated, selecting evaluation indexes and index calculation, and evaluating and displaying the results of English-Chinese translation. Through the index loading, the translation result evaluation index can be loaded. The index calculation is the calculation of the evaluation index of translation results. Translation quality evaluation module: determine the translation effect according to the translation result evaluation index. The algorithm flow chart in the system is shown in Figure 3.

The algorithm steps can be briefly described as follows: (1) preprocessing the translation data corpus to extract semantic vectors (source phrases and target phrases); (2) according to the semantic vector mapping model, realize the semantics of source phrases to target phrases; (3) calculate the translation similarity of different semantic vectors in the same translation environment according to the translation similarity model; (4) select the translation similarity as the feature vector, and add it to the translation decoding to obtain the translation result.

RETRACTED

The feature extraction algorithm maps the optimal context into the translation process in order to achieve the standard extraction of feature context. It is assumed that there are *N* translation contexts in the translation process, in which *K* has class semantic translation, the number of translation contexts is *N*_*i*_, and *K* class semantic translation is represented by probability as *X*_*i*_, where *K* is a set of directional dimension vectors. The translation that can achieve the basic standard translation context through the qualification process is shown in the following formula:

(1) $$\begin{array}{c} \alpha_{i}=\frac{1}{N}\overset{N_{i}}{\underset{j=1}{\sum }}x_{ij}, \end{array}$$

where *α*_*i*_ is the semantic translation context that can be translated, and the expression of the selection process of the best context *α* is as follows:

(2) $$\begin{array}{c} \alpha =\frac{1}{K}\overset{K}{\underset{i=1}{\sum }}\alpha_{i}. \end{array}$$

The expressions suitable for the semantic translation context matrix *S*_*B*_ and the nonsemantic translation context matrix *S*_*w*_ are calculated as follows:

(3) $$\begin{array}{c} S_{B}=\overset{K}{\underset{i=1}{\sum }}\left(\alpha -\alpha_{ij}\right){\left(\alpha -\alpha_{ij}\right)}^{k}, \end{array}$$

(4) $$\begin{array}{c} S_{w}=\overset{K}{\underset{i=1}{\sum }}\overset{Ki}{\underset{j=1}{\sum }}\left(\alpha_{ij}-\alpha \right){\left(\alpha_{ij}-\alpha \right)}^{k}. \end{array}$$

Assuming that *λ* is the optimal context of the semantic context correlation matrix *S*_*w*_^*T*^*S*_*B*_ and *f* is the standard to measure the semantic context correlation, the value of *α* can directly reflect the mapping of the correlation process. The phrase table is another name for the translation model. The phrase table keeps track of bilingual phrase pairs and the likelihood that each pair will be translated. A phrase in statistical machine translation refers to a run of words in a sentence, whether it be in the source language or the destination language, and is not always a phrase in the grammatical sense. The phrase table is a set, and each element in the set provides the following information: lexical translation probabilities, phrase translation probabilities between phrase pairs, source language, target language, and phrase pair probabilities. The meaning of being consistent with word alignment is: if all words in the source phrase *s* are aligned with the target phrase, and this rule is also satisfied in the reverse direction, then (*s*, *t*) is said to be consistent with word alignment, and its formula can be expressed as:

(5) $$\begin{array}{c} \text{AND}\exists t_{i}\in t,s_{j}\in s:\left(t_{i},s_{j}\right)\in \text{Align}. \end{array}$$

When extracting the phrase table, it is necessary to extract all phrase pairs that satisfy the following principles: (1) the extracted phrase pairs satisfy the definition of phrases, that is, they should be consecutive word sequences. (2) There should be no word alignment in the extracted phrase pairs. (3) Any word alignment within a phrase pair cannot exceed any phrase at either end. While extracting phrase pairs, it is more important to estimate the probability table between phrase pairs. The translation probability table mainly includes phrase translation probability, lexicalization translation probability, and lexicalization ordering probability. Translation probabilities for phrases include forward (source to target) and reverse (target to source) translation probabilities. Maximum likelihood estimation is a typical technique for estimating translation probabilities. When calculating the forward phrase translation probability of phrase pair (*s*, *t*), first, calculate how many sentence pairs the phrase pair is extracted from, and denote it as count(*s*, *t*); then, count the total number of all legal phrase pairs count; finally, use pairs for normalization operation to get the forward phrase translation probability; its expression is as follows:

(6) $$\begin{array}{c} p\left(t\left|s\right.\right)=\frac{\text{count}\left(s,t\right)}{\sum_{t_{i}}\text{c}\text{ount}\left(s,t\right)}. \end{array}$$

Lexical translation probabilities include forward and reverse lexical translation probabilities. Lexical translation probability describes the probability of mutual translation between words within a phrase and is also a basic smoothing method. As part of the translation model, the lexical translation probability also has an important impact on the performance of the machine translation system. For a sentence *s* = *w*_1_*w*_2_ ⋯ *w*_*t*_ composed of primitives (“primitives” can be word sequences such as words, words, phrases, etc.), according to the Markov chain, causal hypothesis, in the statistical language model, it is assumed that the occurrence probability of the current word is only related to the previous word, such as when *n* = 3 is given, that is, the probability of a word only depends on the two words in front of it, which is called a 3-gram model, that is, a third-order Markov chain, denoted as trigram. Then, the chain rules are:

(7) $$\begin{array}{c} p\left(s\right)=\overset{i}{\underset{i=1}{\prod }}p\left(w_{1}\cdots w_{i-1}\right)\approx \overset{i}{\underset{i=1}{\prod }}p\left(w_{1}\left|w_{i-1}w_{i-2}\right.\right). \end{array}$$

The parameters of the statistical natural language processing model are counted from the corpus, and the parameter estimation adopts the maximum likelihood estimation method:

(8) $$\begin{array}{c} P_{mle}\left(w_{1}\left|w_{i-1}w_{i-2}\right.\right)=\frac{C_{3}\left(w_{i-2}w_{i-1}w_{1}\right)}{C_{2}\left(w_{i-2}w_{i-1}\right)}. \end{array}$$

Assuming that the random variable obeys the normal distribution, we estimate the parameters of each translation through the probabilistic statistical method. The formula of the normal distribution probability density function is:

(9) $$\begin{array}{c} f\left(t\right)=\frac{1}{\sigma \sqrt{2\pi }}e^{\left(\left(t-\mu \right)/\sigma \right)2}\sigma . \end{array}$$

Dialogue management is the most important part in the process of human-computer interaction. The core content of dialogue management is to guide the human-computer interaction through certain policy control. In the early dialogue systems, the slot filling method is generally used to realize the dialogue management. For example, the galaxy system regards the dialogue process as the filling process of the slot through continuous interaction until the dialogue goal is achieved. The implementation method of this dialogue process is mechanical and inflexible. The Markov decision process is introduced into the dialogue management, and the dialogue process is mapped into a statistical model. The dialogue strategy control is regarded as the process of solving the optimal problem under a certain cost function. The so-called translation similarity model refers to the similarity of two semantic vectors *u* and *v* in the same translation environment. If the similarity of the two semantic vectors *u* and *v* is higher, the semantics of the two semantic vectors *u* and *v* are closer. In this paper, the cosine similarity function is selected to measure the translation similarity between two semantic vectors *u* and *v* in the same translation environment. The expression is as follows:

(10) $$\begin{array}{c} \text{Sim}\left(u,v\right)=\frac{u\cdot v}{\left\|u\right\|\times \left\|v\right\|}=\frac{\sum_{i}\left(a_{i}\times b_{i}\right)}{\sqrt{\sum_{i}a_{i}^{2}\times \sum_{i}b_{i}^{2}}}, \end{array}$$

where Sim(*u*, *v*) is the translation similarity of two semantic vectors *u* and *v* in the same translation environment. Decoding is translation. In the human-computer interactive cooperative translation system, decoding is the process of searching for the best translation using translation model, language model, lexicalization, and order model. Translation word selection method based on user translation history. After the translation template is determined, the variable part in the template needs to be translated. For the case that the same word or phrase has many different translation methods, this paper determines the choice of word meaning by calculating the similarity between all sentences containing the variable in the current user's translation history and the current sentence to be translated. Like many problems in natural language processing, the decoding of machine translation is a structured search problem, and its search space is exponential, so it is impossible to exhaust the entire search space. We need a less complex algorithm to search for the best translation. Based on the automatic postediting technology of machine translation, the machine translation is taken as the source language, and the correct translation modified by each user is taken as the target language. The statistical translation model is trained by the human-computer interaction cooperative system. Before recommending the machine translation to the current user, the machine translation is translated into an auxiliary translation closer to the correct translation by using its own translation model. Thus, the number of postediting operations by the user can be further reduced and improve the efficiency of collaborative translation.

RETRACTED

## 4. Result Analysis and Discussion

In order to ensure the uniformity of the test parameters and the objectivity and validity of the test results, the test parameter types include the following: vocabulary test data, short sentence test data, and long sentence test data. The maximum value of vocabulary contained in the long sentence test data is 100 characters, and the maximum value of words and sentences in the long sentence composition text is 800 characters. In order to ensure that the translation test can be carried out normally and the test results are objective, avoid overfitting, and shorten the gap between the training error and the test error, the gradient descent method is used to set the relevant translation threshold as the intermediate point to stop the iteration process. The translation threshold is shown in Table 1.

From the test samples and test thresholds set in Table 1, it can be seen that in this process, the translation threshold rate can ensure the normal progress of the test, and the set threshold is only the minimum guarantee value. The actual rate value of both translation systems is greater than this value. Therefore, the set rate will not disturb the test results and affect the objectivity of the results. We conducted experiments on the BTEC Chinese English text translation tasks of iwslt2017 (international work shop on spoken language translation) and iws-lt2018, respectively. The translation engine adopts the human-machine interactive collaborative translation system based on artificial intelligence technology developed by us. We extract phrases from the training sets of the two tasks to adjust the parameters of the translation system. Here, the two tasks are called smt07 and smt08, respectively, for convenience. The basic statistics of experimental data are shown in Table 2.

RETRACTED

During training, we use their phrase tables to generate extended sentences on the iwslt2017 and iwslt2018 development sets to extract features and train SVM classifiers. We trained 7 classifiers on the iwslt2017 development set. Six classifiers were trained on the iwslt2018 development set. During the test, we generate extended sentences on the respective test sets, extract the features, and classify the extended sentences with a combination classifier. Finally, human-computer interaction is used to select the best translation result. We take the translation system constructed in this paper as our baseline system; compare the traditional translation machine based translation system with the human translation-based translation system. In the process of human-computer interaction. The user's burden needs to be considered. If the system repeatedly asks questions for a sentence and cannot get the result quickly, it will make the user feel bored, thereby reducing the efficiency of the interaction. The interaction data of users in the experiment are shown in Table 3.

As an illustration, the smt17 challenge contained 493 Chinese sentences, 225 of which were processed using a human-computer interface. With an average of 1.68 interactions per sentence, there were 362 interactions. There were 55 sentences with two interactions, making up 15.2% of the total and accounting for 80.9% of them in total. There were 238 sentences among them with a single interaction, meaning that 65.7% of the total can be reached after just one encounter. From the data, it is clear that consumers have a minimal strain during the human-computer contact process. To decide whether there are phrases in the candidate phrases that have the same semantics as the whole sentence, usually 1 to 2 options are required. The suggested translation system's performance is tested against competing systems in order to confirm its actual performance.  Figure 4 displays the outcomes of weight changes for several types of semantic recognition.

From Figure 4, we can see that for different types of semantic recognition weight changes, the change range of the control weight of the short sentence is 0~0.82, while the change range of the control weight of the long sentence for the word is 0.7~1.07, and the volatility is smaller than that of the short sentence. To further test the advantages of the system at the data level, the change results of the minimum editing distance when the relative entropy takes different thresholds are shown in Figure 5.

RETRACTED

Figure 5 depicts the minimal editing distance change curve for various relative entropy levels between 0.1 and 0.6, respectively. Figures 6 and 7 show, for various systems, the translation accuracy and accuracy of the conventional machine translation system, the human translation system, and the system developed in this research under various adaption indices.

As can be seen from Figures 6 and 7, compared with traditional machine translation system and human translation system, the accuracy and accuracy of the translation system constructed based on this paper are the highest under different adaptation indexes. In a fully automatic machine translation system, the translation results of the system are completed by machine learning alone. The knowledge source used by the system is completely static and cannot be dynamically generated. Compared with the automatic machine translation technology, in the human-computer interaction collaborative translation system, the user can screen, evaluate, and edit the auxiliary translation automatically generated by machine translation until the best translation with the closest result to the human translation is finally obtained. In the collaborative translation system, the template base is established by incremental learning, that is, when the number of sentences that do not match the templates in the existing template base reaches a certain number, the system extracts new bilingual templates from the newly generated translation history and stores them in the system template base. Therefore, the system performance will be continuously optimized with the increase of the use time and the number of people. In order to further verify the performance of the system, the comparison results of recognition tolerance under different systems are shown in Figure 8.

From Figure 8, it is clear that the recognition tolerance analysis of the other two systems and the system developed in this paper shows that the overall recognition effect of the other two systems is not as good as the human-computer interaction collaborative translation system mentioned in this paper. The control effect of the system developed in this paper on the control of words, short sentences, and long sentences is also obvious, indicating that according to the experimental findings, the human-computer interaction cooperative translation system, which is based on artificial intelligence technology, has a translation accuracy range between 95.6% and 98.2%. After human-computer contact and cooperation, the quality of the translated translation improves, and the editing distance between the incorrect translation and the auxiliary translation is reduced, demonstrating the effectiveness of the system and demonstrating its viability. In order to increase the system's translation quality and operational efficiency, research into collaborative translation modes based on human-computer interaction is important.

RETRACTED

## 5. Conclusion

People today must translate between several languages due to the rising frequency of global contact. Large-scale translation demands are difficult to achieve due to the high cost and poor efficiency of human translation, which is why demand for autonomous translation technology is rising steadily. The overall progress in this field is machine translation technology. The translation quality of machine translation is still imperfect after a long period of development, despite the fact that the technology is constantly evolving and maturing. As a result, it is challenging for users to directly use machine translation in situations where there are strict requirements for translation quality. In light of this issue, a novel concept known as collaborative translation mode for human-computer interaction is suggested. This study mainly investigates the machine translation mode for human-machine interaction based on artificial intelligence technology and analyses the model adaption, decoding algorithm, and other aspects of HMI. By addressing the shortcomings of the existing interactive machine translation, it enhances the capability of the collaborative translation system for human-machine interaction and lowers the price of user translation. In this study, an artificial intelligence-based interactive collaborative translation system for humans and machines is built, and its effectiveness is evaluated. According to the experimental findings, the accuracy of the human-machine interactive collaborative translation system based on artificial intelligence technology can reach 98.2% and 95.6%, respectively. The editing distance between the auxiliary translation and the proper translation is reduced, which indicates that the system is successful and demonstrates its viability. The quality of the translated translation is also improved as a result of the human-machine interactive collaboration. As a result, research into collaborative translation modes based on human-computer interaction is important for enhancing system translation quality and operational effectiveness.

## Figures and Tables

**Figure 1:** Schematic diagram of machine translation pyramid.

RETRACTED

**Figure 2:** Human-computer interaction collaborative translation system based on artificial intelligence technology.

**Figure 3:** Algorithm flow chart.

**Figure 4:** Test the weight change of different types of semantic recognition.

**Figure 5:** Change of minimum editing distance when relative entropy takes different thresholds.

**Figure 6:** Changes in translation accuracy under different adaptation indices.

**Figure 7:** Comparison of translation accuracy under different adaptation indices.

**Figure 8:** Comparison of recognition tolerance under different systems.

**Table 1:** Test sample data parameters and translation threshold setting.

Sample parameter type	Minimum length/character	Maximum length/character	Translation threshold
Vocabulary	2	15	20
Short sentence	4	22	15
Long sentence	8 (200)	150 (800)	10

**Table 2:** Statistics of experimental data.

Task	Training set	Development set	Test set	Phrase length limit	Phrase table scale
SMT17	268785 sentences	495 sentences	495 sentences	8	389820 sentences
SMT18	322745 sentences	784 sentences	512 sentences	22	425369 sentences

**Table 3:** Statistics of human-computer interaction data.

Task	SMT17	SMT18
Total sentences	493	515
Interactive sentence	225	329
Total number of interactions	362	488
Average interaction times	1.68	1.89
Interactive successful sentences	162	95

## Data Availability

The data used to support the findings of this study are available from the corresponding author upon request.
